# Analysis of Machine Translation and Post-Translation Editing Ability Using Semantic Information Entropy Technology

This article has been retracted.

**DOI:** 10.1155/2022/5932044

**Published:** 2022-08-18

**Authors:** Siyu Zou

**Affiliations:** School of Foreign Languages, Nanchang Institute of Technology, Nanchang 330000, China

## Abstract

Large-scale corpus application has presented MT with new opportunities as well as challenges in recent years. This study investigates MT and post-translation editing capability using AI technology. The grammar rules of the target language are first examined. Then, a significant amount of data on semantic information entropy are projected, and the semantic Gaussian marginal rectangular window function is obtained. The semantic correlation factors of words are added to the text information entropy and information gain, and the nonlinear spectral properties of adaptive matching semantics are obtained. In this way, it corrects the significant flaw in the way semantic features are extracted using conventional techniques. In order to speed up MT and enhance translation quality, this study proposes automatic post-translation editing to filter those common MT errors that occur frequently and regularly. According to the experimental findings, word translation and segmentation accuracy can both reach 95.27 and 93.12 percent, respectively. In terms of language translation, this approach is accurate and trustworthy. I hope it will serve as a useful source for subsequent research.

## 1. Introduction

Language serves as the primary means of intercultural communication in the information technology era of the twenty-first century, and the process of cultural communication depends heavily on language translation. The development of nations and regions, particularly economic development, depends largely on high-quality translation services [1]. It can not only eliminate language barriers and enable the efficient exchange of information between nations and nationalities, but it can also significantly advance international trade, cultural exchange, and national cohesion. The need for translation services has skyrocketed, the volume of translations has increased quickly, and the range of materials that need to be translated has grown significantly in recent years [2]. MT (Machine translation) technology, which can achieve automatic natural language translation, has been a major research hotspot in the field of AI (Artificial intelligence) for more than 10 years. This is because, when faced with the vast amount of multilingual information, traditional manual translation is far from meeting the needs. One of the core issues in computational linguistics and artificial intelligence is MT [3]. Every advancement in MT research helps us understand human intelligence, language, knowledge, and other issues better. It can also serve as a reference for natural language processing and other problems related to it in other fields. People initially had high expectations for machine translation (MT), held the narrow belief that it would replace human labor, and saw MT as the end result of the translation process without pre- or post-translation editing. The outcome was not good enough [4]. The two main stages of development for MT were rationalism and empiricism. Although the former can analyze, transform, form natural language and describes translation knowledge according to the law of transformation between human extraction and natural language, there are many drawbacks, including a greater challenge in integrating translation knowledge, a lengthy development cycle, and a high labor cost [5]. Additionally, it is crucial to revise and enhance the translation of MT through post-translation editing in order to guarantee its quality and applicability.

The application of large-scale corpus has brought new opportunities and challenges to MT. Technological progress has changed people's view of traditional translation, and the technical characteristics of the translation industry process have become increasingly prominent [6]. More and more language service providers begin to use computer-aided translation tools with translation memory, terminology database and many other functions in the translation process. The traditional translation mode has quietly changed and becomes a human-computer interaction activity. However, while MT is improving its speed, its translation quality has been criticized [7]. There are two main ways to improve the quality of MT translation: ① further improve MT software to improve the quality of the generated text; ② Post-translation editing of the machine translation. There are many translation algorithms, but not every translation algorithm plays the best role in any case, so it is necessary to analyse the running efficiency of each translation algorithm, that is, the running time, to focus on their different advantages and disadvantages in the same situation [8]. Most of the language processing mechanisms created by MT for a variety of natural languages are rudimentary and rely too heavily on manual summarization by linguists, which is unsuitable for machine processing of some linguistic details and prone to the drawbacks of significant translation errors. Translation companies and language service providers are looking for faster translation methods, and post-translation editing based on MT fills the gap between MT and human translation. This study conducts inventive research from the following angles in order to address the aforementioned issues and create a translation model with better generalization capacity:

- Based on the in-depth study of AI technology and MT-related literature, this study constructs an MT model with better generalization ability and higher translation accuracy. In this study, a large number of semantic information entropy data are projected; In the text information entropy and information gain, the semantic correlation factors of words are added, and the nonlinear spectral characteristics of adaptive matching semantics are obtained. In this way, it makes up for the big error of semantic features extracted by traditional methods.
- Aiming at those typical MT errors with regularity and high frequency, this study envisages automatic post-translation editing to filter these typical errors, so as to speed up MT and improve translation quality. Simulation results show that the proposed method achieves a good MT effect and has a good development space.

This study mainly discusses MT and post-translation editing ability. The specific organizational structure is as follows.

## 2. Related Work

Labaka et al. have studied an English MT improvement method based on TFIDF. This method first obtains the information entropy and information gain of the language. On this basis, it integrates the semantic association factors of words and completes the improvement of English MT under the weakening grammar rules [9]. This method is simple, but it has the disadvantage of poor scalability. Starting from discussing the concept of post-editing, Tan et al. analyzed the application and research status of post-editing, summarized the development momentum of post-editing, studied the subject types applicable to post-editing, and put forward practical guidelines to improve the quality and efficiency of post-editing [10]. In order to improve the speed of traditional stand-alone translation algorithms, there are some optimizations for language model query performance. Screen proposed the use of Bloom filters to handle very large-scale language models [11]. But this method compresses the amount of data, which reduces the accuracy. Nguyen et al. avoided repeated queries during query rollback by caching the left and right states of language model queries [12]. Dombrowski et al. combined cache and HASH index to improve query efficiency [13]. But HASH indexes lead to wasted space due to the need for additional free space. Tong and Zhu expanded the amount of training data for under-resourced languages through data augmentation technology, thereby enhancing the generalization performance of neural MT [14]. Xiong et al. believe that translation ability and post-translation editing ability overlap, but they are not the same. Post-translation editing requires three major categories of competence, namely language competence, tool competence and core competence [15]. Xue proposed an improved method for English MT based on semantic features. This method first defines the English semantic features, extracts the essential features of the semantic features, divides the English semantic features into four categories, and completes the improvement of English MT for different categories [16]. This method has strong scalability, but when using this method to improve English MT, it relies too much on the manual summary of language experts and has the disadvantage of large errors in semantic feature extraction. Stymne et al. proposed an Uyghur–Chinese neural MT model for subwords and words, converted the translation unit of a word into a mixed translation unit of words and subwords, used the nonlinear unit of ALU as the neural nonlinear unit of GRU, and then improved the neural MT model [17]. For the micro-evaluation of MT, Pires proposed an effective MT automatic diagnosis method; he studied key technologies such as the macro-evaluation method based on string similarity, the coverage extension of reference translations, and the automatic diagnosis method for monolingual and bilingual [18]. Fernández-Torné and Matamala adopted an improved method of English MT based on semantics and statistics [19]. The method obtains the rules of constraint rule semantics by forming the English model and semantic analysis model and uses the rules to complete the improvement of English MT. The time complexity of this method is low, but it cannot build a more accurate grammar rule base, and there is a problem of poor translation effect.

This study builds an MT model with better generalization capability and higher translation accuracy based on a thorough analysis of AI technology and MT-related literature. In this study, a large-scale language model and translation model are both used simultaneously, with distributed storage and parallel query mechanisms. This serves as the foundation for further research into a full translation and decoding parallelization algorithm. In order to speed up MT and enhance translation quality, this study proposes automatic post-translation editing to filter those common MT errors that occur frequently and regularly. The proposed method has a good MT effect, according to simulation results, and it produces reliable and accurate language translations.

## 3. Methodology

### 3.1. MT Based on AI Technology

Since different cultures make up the complex whole that is human society, the mutual influence and infiltration of different cultures have aided in the advancement and development of human society. In addition to removing language barriers and enabling effective information transfer between nations, high-quality translation services can also significantly advance cross-cultural dialogue, national cohesion, and international trade [20]. With the widespread use of automatic translation on the Internet, MT-which employs computers to translate between various languages-has gradually gained public acceptance and has emerged as a key tool for bridging the gap caused by the natural language barrier. The process of translating one natural language into another on a computer platform is the aim of machine translation (MT). Recent years have seen significant advancements in MT research, particularly in statistical MT. The issue of obtaining a significant amount of fine-grained translation knowledge from sizable corpora is resolved, and it offers a workable remedy for translation optimization under various complex conditions. The online translation decoding stage and offline language model and translation model training stage are the two main divisions of MT statistics. The three main statistical MT system components-translation model, language model, and decoder-will, however, experience computational performance issues when dealing with large corpora, making it challenging for the current single-machine serial translation processing to finish the calculation in a reasonable amount of time. In computer programming, translation is common and crucial [21]. Due to their distinct translation histories, AIMT and external translation are two of the most important elements of translation. The most popular AIMT among them is appropriate for element sequences with a limited amount of data because it completely stores the data to be arranged in memory before translating it in accordance with their own translation rules. Translation memory and terminology databases are helping the MT system develop in an integrated manner as a result of the quick development of globalization, information technology, and computers as well as their extensive, all-encompassing, and in-depth application in a variety of fields. The pure MT output is no longer the default post-translation editing object because the trained MT system is more intelligent, interactive, and adaptable. The translation process can be seen as a process of transformation at different levels: semantics-syntax-phrase-word. Of course, the lower the level, the less difficult it is to translate. However, the differences in languages determine that translation cannot always be carried out at the lowest level, and the fuzziness and ambiguity of language force us to consider the lower level components at a higher level.

In the usual decoding process, the translation of a short essay often requires millions of queries to the language model, and the queries to the translation model are close to this order of magnitude. Therefore, in the process of real-time online translation, the query efficiency of huge translation model tables and language model tables has become the main bottleneck affecting the performance of online translation decoding process. At present, most models do not make use of deeper structural information such as syntax and semantics, so it is difficult to solve the problem of long-distance word order adjustment in translation. Moreover, the generated translation often does not conform to the grammar of the target language, especially for Chinese and English, two languages with big structural differences. Post-translation editing of MT refers to the processing and modifying the original MT output according to certain purposes, such as correcting language or format errors to improve the accuracy and readability of machine-translation output. Post-translation editing can generally be divided into light post-translation editing and full post-translation editing. Due to the unreliability of MT quality, post-translation editing has become an indispensable link in MT to improve translation quality, which directly determines the quality, speed, and cost of translation. Post-translation editing ability includes four sub-abilities: general ability, technical ability, editing ability, and strategy ability. General abilities include language ability, subject knowledge, cross-cultural ability, literature retrieval, analysis ability, etc. The development of post-translation editing is always closely related to the development of MT, which is the foundation of post-translation editing. This study divides post-translation editing ability into three dimensions: cognition, knowledge, and skills, which are the basic level, the subject level and the realization level. The relationship among the three dimensions is shown in Figure 1.

The wisdom crystallization of the ideal fusion of “artificial” and “intelligent,” AI products are cross-era high-tech, intelligent, and humanized mechanical products. The exponential growth of AI has led to an endless stream of new machine translation (MT) systems and tools, and the interplay between MT and human translation is beginning to generate more and more discussion. It is impossible to separate the advancement of AI technology from the advancement of AI products. The reason AI products are constantly being revised, updated, improved upon, and upgraded is due to the rapid and steady development of AI technology. Using MT of a computer to automatically convert natural language has emerged as a significant research area with the rapid development of AI and natural language technology. The advancement of computer technology, which is the technology created by the former, is necessary for the advancement of AI technology. With the rise of AI, globalization, networking, and information technology, there has been an increase in demand for various language services on the global market. Language service providers started to use MT and post-translation editing mode to satisfy this wide range of demand. Realizing the balance between translation quality and efficiency, they switched from human-assisted machine translation to machine-assisted translation. According to the research methods used, MT research can be categorized as rule-based MT, case-based MT, and statistical-based MT. The working environment for translation has changed as a result of the growth of the translation market and the advancement of translation technology, and it will become less common for MT to produce the initial translation. An integrated translation environment for translators is created by combining a translation management system and computer-aided translation (CAT) with “translation memory” technology as its core. Direct insertion translation, Hill translation, simple choice translation, heap translation, bubbling translation, quick translation, merge translation, and cardinal translation are some of the subcategories of translation. All of these translation algorithms can translate data or records and produce the effect of simple searching, but each translation algorithm uses a different data processing method in practice.

### 3.2. MT and Post-Editing Capabilities

The training method has the flexibility to add characteristic functions at will, and each characteristic function has associated weights. Based on this approach, this study defines a loss function for translation model training. In this manner, the particular evaluation criteria can be directly addressed during the training process of such models. The log-linear model is frequently used in statistical MT modeling as a special case of discriminant training. The original noise channel model is a special case of the log-linear model. In order to enhance MT, this study analyses the semantics of the input source sentences first. Then, using the provided grammar conversion rules, it determines the relationships between the source sentence phrases and the corresponding target language phrases. On this foundation, semantic blocks are employed to choose and combine the translation of the phrase sets, and the target language's output sentences are created to finish MT. From the bilingual corpus, all synchronization rules and their weights are extracted, counted, and stored in the translation model table. Decoding is the process of figuring out each target word's conditional probability when it is output in a known part. The performance of the decoding algorithm, a crucial component of statistical MT research, directly influences the final translation's quality and effectiveness. The hierarchical phrase-based decoding procedure resembles the conventional parsing procedure. It continuously stipulates source language sentences using synchronous grammar rules from bottom to top, and pruning is used in conjunction with the stipulation process to avoid creating too many combinations of upper nodes. The output operation is carried out by the decoder by converting the intermediate vector produced by the encoder to the target vector. The encoding process ends and the decoding stage begins if the encoder receives the end identifier of the source input text. The decoder framework is shown in Figure 2.

In the process of optimizing MT, the grammar rules of the target language are analyzed, and a large number of semantic information entropy data are projected after obtaining the semantic Gaussian marginal rectangular window function. The way to solve the problem of ordering and data sparseness is to introduce syntactic information on the basis of the phrase model. However, both the method of introducing unilateral syntactic information and the method of introducing bilateral ten-day syntactic information are faced with the problems of non-syntax of phrases and the heterogeneity of bilingual syntactic structures. Through the improvement, the running process is shortened by half by taking out the two maxima, which effectively improves the efficiency and the iteration time compared with the common translation algorithm. Therefore, the application of this improved method in selecting translation algorithms is necessary and effective. The translation errors of MT mainly come from the logical and structural errors of complex sentence patterns, such as errors in ellipsis, reference, and juxtaposition. Wrong choice of word meaning, isolated words, wrong transformation of syntactic structure, wrong form, etc. Specifically, high-quality post-translation editing needs to pay attention to the existence of semantics, grammar, pragmatics, terminology, spelling, punctuation, symbols, numbers, formatting errors, additions, omissions, ambiguities, consistency, cultural conflicts and so on.

It is assumed that *T* represents the source sentence set, *T*_*i*_ represents the segmented source sentence, and *j* represents the translatable type of the source phrase sequence. Then use formula (1) to obtain the source sentence phrase and the corresponding phrase link:

(1) $$\begin{array}{c} D_{ij}=\frac{R_{*}}{D_{n}}\cdot \left(T\times T_{i}\right)j. \end{array}$$

In the formula, *R*_*∗*_ represents the given grammar conversion rule, and *D*_*n*_ represents the semantic block. Hypothetically, the main semantic role is represented by *∂*(*t*); the recognition of prepositional phrases is represented by *p*(*o*). Then use formula (2) to select and combine the translations of the phrase set:

(2) $$\begin{array}{c} S_{ww}=\frac{w_{i}\cdot \partial \left(t\right)}{p\left(o\right)}*SC\left(o\right). \end{array}$$

The word's modifier is represented by *w*_*i*_ in the formula, and the number of semantic blocks built in accordance with the grammar library is represented by *SC*(*o*). Assume that *γ*^*∗*^ represents the value of the entry in various grammatical formats and that *H* represents any dictionary entry. Φ^‴^ represents the extracted source sentence feature. Utilize formula (3) to finish MT improvement:

(3) $$\begin{array}{c} WE_{\gamma }=\left(\frac{\Phi^{\prime \prime \prime }•H}{\gamma^{*}}\right)\left(\frac{\left(F\right)\cdot S_{ww}}{D_{ij}}\right)\vartheta_{*}. \end{array}$$

In the above formula, *ϑ*_*∗*_ represents the redundancy of knowledge. In the initial stage of encoding, the Embedding layer of the encoder will encode all the vocabulary *x*_*i*_(*i* ∈ *n*) of the source input text and convert it into the word vector expression shown in the following formula:

(4) $$\begin{array}{c} W^{i}\in R^{\left|V\right|}\;i=1,2,3,\ldots ,T, \end{array}$$

(5) $$\begin{array}{c} W^{i}=\left[n_{1},n_{2},n_{3},\ldots ,n_{m}\right],\;n_{i}\in R. \end{array}$$

Among them, the source language vocabulary size is *V*.

A core problem of statistical MT is to define a statistical translation model, that is, the probability *P*(*t|s*) of a source language sentence *s* translated into a target language sentence *t*. Hierarchical phrase-based statistical MT is described using a log-linear model. Given a source language sentence, define its translation $\hat{t}$ as follows:

(6) $$\begin{array}{c} \hat{t}\left(s\right)=\underset{t}{\arg\;\max P\left(t|s\right)}=\underset{t}{\arg\;\max}\prod_{i=1}^{m}{\left[\varphi_{i}\left(t,s\right)\right]}^{\lambda_{i}}. \end{array}$$

Among them, *φ*_*i*_(*t*, *s*) is the characteristic function whose value is the probability, and *λ*_*i*_ is the weighting coefficient of *φ*_*i*_. Taking the logarithm of both sides of the equation, we get

(7) $$\begin{array}{c} \hat{t}\left(s\right)=\underset{t}{\arg\;\max}=\sum_{i=1}^{m}\lambda_{i}h_{i}\left(t,s\right), \end{array}$$

(8) $$\begin{array}{c} h_{i}\left(t,s\right)=\ln\;\varphi_{i}\left(t,s\right). \end{array}$$

Among various feature functions, the two most important feature functions are the translation model and the language model. Using the syntactic information to guide the ordering problem of the target language generation process, the ternary structural model is defined:

(9) $$\begin{array}{c} h_{3}\left(A\right)=\log\prod_{i=1}^{K}p\left(R_{i}\left[T\left(e\right)\right]|R_{i-1}\left[T\left(e\right)\right],R_{i-2}\left[T\left(e\right)\right]\right). \end{array}$$

The text category to be translated is defined as the information source, and the relationship between word information entropy and word weight is determined by the information gain relationship between the category information entropy of the training data set and the conditional entropy of words in the document category to be translated. Then it is expressed by the following formula:

(10) $$\begin{array}{c} {\text{Weight}}_{tfidf}\left(t_{i}\right)=\frac{tf\times idf\;\times IG\left(C,t_{i}\right)}{p\left[cj\right]*\ell \left(i,t\right)}, \end{array}$$

where *IG*(*C*, *t*_*i*_) represents the training data set; *ℓ*(*i*, *t*) represents the conditional entropy of the words in the category of documents to be translated; *p*[*cj*] represents the conditional information entropy of the words.

In order to achieve high-quality post-translation editing, it is necessary to obtain the translated text with correct semantics, no omissions and additions of information, revise the offensive or inappropriate content in the target culture, and pay attention to the problems of grammar, syntax, terminology, punctuation, and format. A synchronization rule consists of a prescribed symbol and a pair of equivalent symbol strings of the source language and target language, in which the non-terminators in the source language string and the target language string correspond one to one. Because the synchronization rule is automatically extracted from bilingual corpus, in order to prevent too many synchronization rules, it is generally stipulated that a synchronization rule should contain at most two non-terminators. Based on the phrase model, this study introduces the concept of the meta-structure group to identify syntactic and non-syntactic phrases. Using syntactic information to study the ordering of phrases in the process of translation, the concept of structural model based on the meta-structural group is put forward, and the related theories and algorithms for studying structural model are expounded. At the same time, an intermediate intonation order model is proposed to reduce the degree of structural heterogeneity between the target language and the source language and improve the translation quality.

## 4. Result Analysis and Discussion

This chapter gives the experiment of this model and its application to MT and build an optimized platform of MT on Windows platform. In the experiment, the feature training set based on the phrase is the same as the structural model training set based on meta-structure. Adopt the test set of NIST T04 Chinese-English evaluation as the development set; The test set of NIST05 Chinese-English evaluation is used as the test of this experiment. The decoder adopts completely consistent decoding algorithms, data sets, and parameters, and does not adopt any performance optimization aiming at the characteristics of natural languages. The purpose of this is to ensure that under the premise of basically consistent BLEU scores, the influence of language-related optimization on performance is eliminated, so as to compare the computing performance of different systems.  Table 1 shows the performance of the input translation system in some special linguistic categories of source languages.

Using the obtained training set, a data set of 500 sentences is extracted, which is used as the weight training of the structural model, and the rest of the data is used as the training set of the feature function.  Figure 3 shows the growth rules of the three models under different scale corpora.

In the process of using this algorithm for MT, the semantic correlation factors of words are added to the middle of the text information entropy and information gain, and the nonlinear spectral characteristics of adaptive matching semantics are obtained, thus ensuring the overall effectiveness of this algorithm for MT. As a comparison, in the experiment, the performance upper limit of the sentence-level translation fusion method is calculated on the development set and the test set respectively. For sentence-level evaluation, we smooth BLEU by adding a small value to the N-gram count. The quality of the fused translation is evaluated by BLEU-4. The evaluation tool used is mteval-v11b.pl, and the parameters are the default parameters.  Figure 4 shows the performance comparison results between the system with intermediate tone sequence restriction and the baseline system.

The experiment shows that although the performance of the system with intermediate tone sequence restriction is improved compared with that of the baseline system, the difference is not obvious. The reason is that in the process of translation, the number of phrases that can be used in the translation of sentences with short lengths is relatively small. It is assumed that any word order between phrases in the process of translation can be taken into account, so that the language model can almost be competent for word order adjustment in the process of translation.  Table 2 shows the experimental results on the development data set.

English MT optimization experiments are conducted using the algorithm presented in this paper and the other two algorithms. Utilize the comparison results to gauge the accuracy of two different English MT algorithms by comparing the word and text segmentation accuracy of the two algorithms. The comparison of the word accuracy rates of various algorithms is shown in Figure 5.  Figure 6 displays the comparison outcomes of the segmentation precision of various algorithms.

The analysis leads to the conclusion that this algorithm produces English MT optimization with a higher accuracy than the comparison algorithm. This is primarily due to the fact that English grammar rules are first examined, a semantic Gaussian marginal rectangular window function is obtained, and a significant amount of information entropy data for English semantics are projected as part of the process of using this algorithm to optimise English MT; therefore, the accuracy of English MT optimization by this algorithm is effectively guaranteed. In the experiment, for each sentence in the source language in each input system, we obtain a set of 10-best candidate translations. If an input translation system or a sentence cannot provide enough candidate translations, we will supplement the 10 candidate translations by repeating the best translation. Finally, the scores of candidate translations from the same input translation system for each source language sentence are normalized. In order to test the effect of rule filtering, we randomly selected 5000, 10000, 15000, and 20000 syntax tree pairs from the training set, and conducted four experiments to compare the BLEUScore scores of the model with and without rule filtering under the same decoding system, as shown in Figure 7.

It can be seen that when the filtering constants of both languages are set to 4, the BLEU Score of the system does not decrease obviously. In fact, the overall load of the cluster is not very high when the decoder in this study performs translation under 80 threads. Therefore, if the concurrency continues to be improved, there is still room for improvement in translation speed in theory. The experimental results in this chapter show that the accuracy of word translation and segmentation can reach 95.27% and 93.12% respectively. At the same time, its post-translation editing ability has been enhanced, and language translation using this method has certain accuracy and reliability.

## 5. Conclusions

MT technology has advanced significantly in recent years, which has been acknowledged by the translation industry and customers, and has made it an essential component of an effective translation process. This progress has been made possible by the development of software technology, the appearance of new algorithms, and improvements in computer performance. Additionally, post-translation editing proficiency is a recent research area in the field of translation studies. This study builds an MT model with better generalization capability and higher translation accuracy based on a thorough analysis of AI technology and MT-related literature. The target language's grammar rules are first examined. Then, a significant amount of data on semantic information entropy are projected, and the semantic Gaussian marginal rectangular window function is obtained. The semantic correlation factors of words are added to the text information entropy and information gain, and the nonlinear spectral properties of adaptive matching semantics are obtained. Additionally, the entire large-scale language model and translation model utilize parallel queries and distributed storage simultaneously. This serves as the foundation for further research into a full translation and decoding parallelization algorithm. In order to speed up MT and enhance translation quality, this study proposes automatic post-translation editing to filter those common MT errors that occur frequently and regularly. According to simulation results, word translation and segmentation accuracy can be as high as 95.27 percent and 93.12 percent, respectively. Its capacity for post-translation editing has also been improved. When MT processing is based on a large corpus, the proposed method achieves a good MT effect and good system scalability. This model has some theoretical and practical significance and can offer some recommendations for further research in related fields. The research in this study still has some shortcomings though. The following step entails enhancing system performance, system structure, and contributing to the translation community.

## Figures and Tables

**Figure 1:** Three-dimensional model of post-translation editing ability.

**Figure 2:** Decoder framework.

**Figure 3:** Changes of models under different scale training sets.

**Figure 4:** Comparison results of system performance.

**Figure 5:** Comparison of word accuracy for translation by different algorithms.

**Figure 6:** Segmentation accuracy of translation by different algorithms.

**Figure 7:** Comparison of BLEU score before and after rule filtering.

**Table 1:** Performance of translation system in linguistic category.

Linguistic category	Sys_1	Sys_3	Sys_5
*Lexical level*			

Ambiguous words	0.526	0.435	0.627
Idiom	0.184	0.177	0.298
*Phrase level*			

Subject-predicate collocation	0.324	0.342	0.374
Verb-object collocation	0.421	0.389	0.436
Quantifier phrases	0.458	0.457	0.481

**Table 2:** Experimental results on the development data set.

Input and fusion translation	BLEU-4
*Input translation system*	

Sys_l	0.3321
Sys_2	0.2901
Sys_3	0.2806
Sys_4	0.2907
Sys_5	0.2746
*Sentence-level translation effects*	

wMBR-BLEU	0.3415
wMBR-BLEU (Sys_2, 3, 4, 5)	0.2928
wMBR-NIST	0.3406
wMBR-TER	0.3254
wMBR-GTM	0.3367
wMBR-SNR	0.3369
MBR-BLEU	0.3354
Con_wMBR-BLEU	0.3361
Multi-features	0.3398
Sen-level upper bound	0.4114

## Data Availability

The data used to support the findings of this study are available from the corresponding author upon request.
